The article "A Corpus-Driven Study on Three Elements of Third Personal Pronoun Endophora in English Abstracts of Chinese and Foreign Theses" was retracted in 2023. Reasons: unreliable results or conclusions; concerns about the data; concerns about the peer review; concerns about the citations.

# A Corpus-Driven Study on Three Elements of Third Personal Pronoun Endophora in English Abstracts of Chinese and Foreign Theses

**DOI:** 10.1155/2022/5981285

**Published:** 2022-03-25

**Authors:** Yuxiao Luo

**Affiliations:** Zhongshan Institute, University of Electronic Science and Technology of China, Zhongshan 528402, Guangdong, China

## Abstract

The corpus is applied to compare and analyze three elements of the third personal pronoun endophora in English abstracts of Chinese and foreign theses. It is discovered that there is no significant difference in the total frequency of third personal pronoun endophora used by Chinese and foreign masters, but there is a significant difference in three elements of third personal pronoun endophora. Native Chinese-speaking masters tend to choose “it” as the anaphor, while native English-speaking masters are inclined to select “them” as the anaphor; antecedents used by native Chinese-speaking masters are mostly consistent with keywords of theses, while antecedents used by native English-speaking masters are rarely consistent with keywords of theses; distances between antecedents and anaphors set by native Chinese-speaking masters are much longer than those set by native English-speaking masters. These findings are beneficial for Chinese masters in terms of better understanding the writing conventions of English abstracts of foreign theses and further improving the language quality of English abstracts in their theses.

## 1. Introduction

Endophora refers to the phenomenon that writers make use of words or phrases to substitute previous or subsequent elements. Endophora seems to be a simple language phenomenon, but actually it not only shows the substitution relation in grammar but also displays the coreferring relation in semantics. Moreover, endophora, as a cohesive means, plays the main constraint on cohesion. Halliday pointed out that anaphors are mostly enacted by personal pronouns [1]. Haiyan LU comparatively analyzed the usage of personal pronouns in general English writing by native Chinese-speaking students and native English-speaking students, and discovered that native English-speaking students tend to choose third personal pronouns as anaphors, while native Chinese-speaking students are inclined to select first personal pronouns to replace complicated and redundant antecedents [2].

In recent years, some Chinese and foreign studies have focused on comparing personal pronoun endophora in English sentences or general English discourses written by native Chinese-speaking students and native English-speaking students. According to Helen and Renate, it is learned that all types of personal pronouns are used as anaphors in general English writing, while in academic English writing, third personal pronouns rather than first and second personal pronouns are preferred [3]. However, the study on third personal pronoun endophora in academic English discourses is relatively rare. Compared with first or second personal pronouns, third personal pronouns not only follow the economic principle of language as they avoid repetitions of complicated antecedents, but also play the role of cohesive means as their comprehension relies on the discourse context. Therefore, third personal pronoun endophora is both a textual language phenomenon and a textual cohesive tool. It is currently a research topic in the spotlight for comparing and analyzing third personal pronoun endophora in academic English writing written by native Chinese-speaking students and native English-speaking students.

This paper employs the tool of corpus to study thirdpersonal pronoun endophora in English abstracts of Chinese and foreign theses. On the basis of the analysis of similarities and differences in third personal pronoun endophora, it is expected to help Chinese masters better understand the writing conventions of English abstracts of foreign theses and to further improve the language quality of English abstracts in their theses.

## 2. Theoretical Framework

According to Halliday, endophora is complicated in that it needs to refer to some elements that have appeared or will appear in the discourse so as to make the whole discourse coherent. When the reference of an element is used to refer to its previous element in the discourse, this phenomenon is called anaphora; when the reference of an element is used to point to its following element in the discourse, this phenomenon is named cataphora [1]. In his dissertation, Jiangli XU claimed that anaphors and antecedents are two inherent elements of anaphora and cataphora [4]. Michael Strumpf demonstrated that anaphors in discourse are mostly expressed by objective third personal pronouns instead of subjective first and second personal pronouns [5]. Forms of personal pronouns consist of subject case form, objective case form, possessive determiner form, possessive pronoun form, and reflexive pronoun form. Compared with other forms, the possessive pronoun form owns double antecedents. For example, “hers” may have the antecedent of “Mary” and the antecedent of “book”. Hua WANG described that those forms of third personal pronoun anaphors are as follows: “He,” “His,” “Him,” “Himself,” “She,” “Her,” “Herself,” “It,” “Its,” “Itself,” “They,” “Their,” “Them,” and “Themselves” [6].

Antecedents in the discourse are generally served by nouns or noun phrases. Since the combination of nouns or noun phrases is infinite, the identification of antecedents is a complicated procedure. Chomsky attempted to propose a series of explanatory rules at the sentential level about antecedents' identification with the aid of the c-command theory of transformational grammar [7]. On the basis of the node analysis and tree-diagram presentation, Levinson claimed that antecedents that have a coindexed relation with anaphors can be identified in the discourse smoothly [8]. Fukumura also adopted c-command as the core idea and claimed that third personal pronouns usually have a coreferring relation with the definite noun phrase in independent sentences [9]. For instance, “Mary thinks she has been late.” If this sentence is an isolated sentence, the third personal pronoun “she” will definitely be regarded as a variable bound by the definite noun phrase “Mary.”

It is clear that Chomsky and Fukumura are restricted to the syntactic level. H.G. Widdowson strode the syntactic node to control the jurisdiction level and confirmed anaphora in discourses by analyzing the semantic characteristics of anaphors and antecedents [10]. However, his method requires a lot of time and energy to analyze the semantic features of third personal pronouns and noun phrases. In order to pursue the labor-saving principle, Levinson and Yan HUANG have raised the antecedent confirmation to the pragmatic level by analyzing partial interpretations, disjoint hypotheses, and salient information interfaces of the coreferring relation [8, 11], but two scholars never touch upon readers' cognitive motivation in the process of discourse comprehension. Ariel and Yulong XU classified anaphors into accessibility levels from the cognitive perspective, and they maintained that pronouns belong to high accessibility markers in that pronouns are closely related to the context in which short-term memory usually works [12, 13].

In comparison to anaphora, the reason why cataphora has not been extensively explored by scholars lies in its rareness. Halliday holds that cataphora is a special linguistic phenomenon which is often discovered in rhetorical or literary writing [1]. For instance, “Through their fiction, the Brontes consider Victorians' treatment and understanding of animals, as well as the human implications and consequences of cruelty.” In this instance, the antecedent “the Brontes” appears after the anaphor “their”, so this phenomenon is genuine backward anaphora. In addition to western scholars, Chinese scholars also make great efforts to investigate cataphora. Through analyzing materials, Yuan GAO and Canlong Wang discovered that although there indeed exists a third personal pronoun cataphora in news titles or subtitles, its application in English writing is still rare [14, 15]. For example, “It may not be great, but Footstep is not that bad”. The anaphor “it” and the antecedent “Footstep” are coindexed in this news title. Therefore, in this research, much attention will be paid to the analysis and discussion of third personal pronoun anaphora instead of cataphora.

Those mentioned researches related to the third personal pronoun endophora indicate that endophora confirmation procedures in discourses should integrate all levels to form a comprehensive endophora confirmation principle. Specific procedures of endophora identification proposed by the author in this paper are as follows:

1. The first step is to seek out the current topic before the anaphor. In the process of topic searching, pronouns are considered as high accessibility markers, so their antecedents are current topics.
2. The second step is to judge whether the anaphor and the current topic are identical in semantic features or not. If they are identical, they have a coreferring relationship; if they are not identical, they do not have a coreferring relationship.
3. The third step is to infer previous and subsequent antecedents based upon contexts at a pragmatic level, and specific contexts are of great importance to identify antecedents.

## 3. Research Design

### 3.1. Research Questions

Three research questions will be answered:

1. What are the similarities and differences in the total frequency of third personal pronoun endophora in the English abstracts of Chinese and foreign theses?
2. What are the similarities and differences in three elements including anaphors, antecedents, and distances used by native Chinese-speaking masters and native English-speaking masters?
3. What are the underlying reasons for discrepancies in the total frequency and specific usage of third personal pronoun endophora applied by Chinese and foreign masters?

### 3.2. Research Instruments

240 English abstracts of Chinese theses are selected from CNKI (China National Knowledge Infrastructure) and 240 English abstracts of foreign theses are selected from PQDT (ProQuest Dissertations & Theses) respectively. CNKI and PQDT are outstanding representatives of Chinese and foreign academic resource databases. AntConc software is applied to transform 480 English abstracts into a corpus. Those English abstracts with more than 100,000 words cover the disciplines of history, literature, sociology, and anthropology. With the aid of concordance, word list, file view, collocates, and other functions in AntConc software, relevant contexts of third personal pronoun anaphors are retrieved. On the basis of the “Hit” column on the left side of the software, the author annotated and analyzed three elements, including anaphors, antecedents, and distances.

### 3.3. Research Procedures

Procedures of data collections consist of three steps:

1. The first step is to automatically search “He,” “His,” “Him,” “Himself,” “She,” “Her,” “Herself,” “It,” “Its,” “Itself,” “They,” “Their,” “Them,” and “Themselves” as third personal anaphors in the corpus.
2. The second step is to artificially analyze the consistency of semantic components between current topics and third personal anaphors by applying the specific pragmatic context and the reader's cognitive capacity. Then the author marks the antecedent as “1” (1 means the antecedent is consistent with keywords of the thesis), and “2” (2 means the antecedent is inconsistent with keywords of the thesis).
3. The last step is to measure the number of words between anaphors and antecedents and consider the distance as the third element, except for anaphors and antecedents.

## 4. Data Analysis and Discussion

### 4.1. Frequency of Third Personal Pronoun Endophora

As endophora is divided into anaphora and cataphora, the total frequency of third-personal pronoun endophora in this research has been counted by the summation of anaphora and cataphora. In 240 English abstracts written by native Chinese-speaking masters, the total frequency of third personal pronoun endophora is 1329, in which there are 1258 anaphora examples and 71 cataphora examples. In 240 English abstracts written by native English-speaking masters, the total frequency of third personal pronoun endophora is 952, of which there are 899 anaphora examples and 53 cataphora examples. In order to test if there exists a significant difference in the frequency of third personal pronoun endophora used by Chinese and foreign masters, the author made use of the Chi-square test in that it mainly deals with the 2 × 2 table for testing the significant difference.

Because of *n* > 40 and an expected count >1, the result of continuity correction^b^ is emphasized in Table 1. The Sig. value of continuity correction^b^ is 0.889, which is much larger than 0.05, hence there is no significant difference in the frequency of third personal pronoun endophora. In other words, both native Chinese-speaking masters and native English-speaking masters tend to apply third personal pronouns to refer to antecedents that appear in the previous or subsequent discourse.

In CNKI and PQDT, the frequency of third personal pronoun anaphora in the disciplines of history and literature accounts for the largest proportion. In CNKI, the cumulative percent in the two disciplines is 58.3%, and in PQDT, the cumulative percent is 65.9%. Masters who major in the disciplines of history and literature are inclined to employ the third personal pronoun endophora. The reason is that the discipline of history mostly involves historical figures, events, and places, and the discipline of literature frequently consists of characters, most of which are proper nouns. When Chinese and foreign masters refer to proper nouns that have appeared in English abstracts, they would like to make use of third personal pronouns to replace redundant antecedents. Only in this way, can the purpose of following the economic principle of language and guaranteeing discourse coherence be achieved.

  Eg1. Based on close reading and text analyses of about 40 historical novels published around 1962, this thesis investigates the differences between these novels, as well as their values and limitations, and demonstrates the profound impact of two of Chen Xiang-he's novels on Chinese literature (sentence from the discipline of literature in CNKI).
  Eg2. This thesis broadly analyzes the principles of Dante's aesthetic in the poem while analyzing the Sibyl, the Hanged Man, and the Prajapati for their relevance to Eliot's aesthetic theory (sentence from the discipline of literature in PQDT).
  In two instances, the third personal pronoun “their” is the economic and succinct anaphor, but “40 historical novels published around 1962” and “the Sibyl, the Hanged Man, and the Prajapati” play the roles of complex and lengthy antecedents. Anaphors acted by third personal pronouns can not only make language succinct in form but also benefit readers in comprehension. That's why third personal pronoun endophora accounts for such a large proportion of the total, no matter in CNKI or PQDT. Both Chinese and foreign masters pay attention to the economic principle of language and focus on the least amount of effort in language and the greatest effect in communication. They tend to apply third personal pronouns in English abstracts so as to reduce complicated and redundant antecedents.
  With the aid of AntConc software and SPSS, 71 genuine cataphora cases were discovered in 240 English abstracts selected from CNKI, and 53 genuine cataphora cases were found in 240 English abstracts selected from PQDT. The author concludes that there exist two types of antecedents. The first type of antecedent is the infinitive form like “to describe…” and the second type of antecedent is the that-clause, like “that the history of Yingzhou Fu has a…“. There is only one type of third personal anaphor. It is the third personal pronoun, “it”. Summarized patterns and specific examples of cataphora in English abstracts written by native Chinese-speaking masters and native English-speaking masters are as follows:
  It is +adj. (like impossible/necessary/…) + to do
  Something makes it + adj. (like significant/important…) + to do
  It is +v-ed (like argued/published/…) + that-clause
  It is +adj. (like significant/important…) + that-clause
  Something makes it + adj. (like significant/important…) + that-clause
  Eg3. It is not normal to do research that associates preschool teachers with professional gender segregation (sentence from the discipline of sociology in CNKI).
  Eg4. Through comparisons of the Broome County Department of Social Services end-of-year caseload reports of 2005 and 2010, it is clear that the number of caseloads has approximately doubled during this time period (sentence from the discipline of sociology in PQDT).
  Eg5. Secondly, the disunity among Jewish organizations made it difficult to put them together as one voice to defend against the destruction of European Jews (sentence from the discipline of literature in CNKI).
  Eg6. To sum up, a comparative study of these two books makes it clear that human beings can only build an ecological society by building a harmonious relationship with nature (sentence from the discipline of literature in PQDT).

After analyzing and discussing third personal pronoun anaphora and cataphora in English abstracts selected from CNKI and PQDT, it is concluded that the usage of the third personal pronoun endophora in English abstracts of theses should be encouraged. On the one hand, third personal pronouns, unlike first or second personal pronouns, are more objective, therefore they are in concordance with the objectivity of theses. On the other hand, the central idea of endophora is to use shorter language representations to substitute longer antecedents. Hence the phenomenon of endophora is the inevitable result of language objectivity and language economy.

### 4.2. Three Elements of Third Personal Pronoun Endophora

In order to test if there is a significant difference in the usage of three elements, including anaphors, antecedents, and distances, used by native Chinese-speaking masters and native English-speaking masters, the author performed an MNOVA test on three elements. The MNOVA test mainly deals with the relationship between two or more fixed factors and various dependent factors. However, according to statistical principles, before the MNOVA test is conducted, the test of homogeneity of variances has been accomplished. As the Sig. value of the test of homogeneity of variances is 0.000, which does not meet the standard of homoscedasticity, in the MNOVA test, “Tamhane's T2” below the line of equal variances not assumed is emphasized. Sig. values in Table 2 show that there exists a significant difference in the usage of anaphors, antecedents, and distances of third personal pronoun endophora used by Chinese and foreign masters.

In terms of anaphors used by Chinese masters, the anaphor “it” has the largest number of 97 in history, the largest number of 93 insociology, and the largest number of 87 in anthropology. The anaphor “it” used by native Chinese-speaking masters is frequently to describe some proper nouns. With regard to anaphors used by foreign masters, the anaphor “their” has the largest number of 70 in history, the largest number of 75 in sociology, and the largest number of 63 in anthropology. The anaphor “they” used by native English-speaking masters is frequently to depict some social spotlights. There are significant differences between the usage of anaphors in the discipline of literature and the usage of anaphors in the other three disciplines. In English abstracts written by Chinese masters, the frequency of the anaphor “it” is the highest in the disciplines of history, sociology, and anthropology, while the frequency of anaphor “his” is the highest in the discipline of literature. In English abstracts written by foreign masters, the highest frequency of anaphor in the disciplines of history, sociology, and anthropology is “they,” while the highest frequency of anaphor in the discipline of literature is “her.”

It is discovered that Chinese and foreign masters majoring in the discipline of literature tend to prefer the third personal pronoun, “his” or “her,” which is determined by professional characteristics. The discipline of literature mostly covers proper nouns for characters in works of literature. In order to avoid cumbersome repetitions of proper nouns, Chinese and foreign masters will use third personal pronouns. As the other three disciplines mostly involve proper nouns and social spotlights, Chinese and foreign masters would like to choose “it” or “their” to replace antecedents in English abstracts for achieving the objective purpose.

At the mention of antecedents applied by native Chinese-speaking masters and native English-speaking masters, there are significant differences in the usage of antecedents among disciplines. In English abstracts, antecedents used by Chinese masters are mostly consistent with keywords of the thesis, but antecedents used by foreign masters are mostly inconsistent with keywords of the thesis. Compared with native Chinese-speaking masters, native English-speaking masters are more inclined to direct readers to experience the whole theme of the thesis rather than simply highlight the topic of the thesis by using repetitions. This difference is traced back to discrepant mindsets and is consistent with the research conducted by Frauen and Shuneng LIAN. According to two scholars, the mindset of Chinese masters displays holistic and inductive characteristics, while the mindset of foreign masters shows analytic and deductive features [16, 17]. The fundamental difference between Chinese and foreign mindsets lies in the perceptual thinking model and the reasonable thinking model. The former employs images to organize perceptual materials so that integral characteristics are portrayed. The latter makes use of logic and reasonable thinking to explore the essence and internal connections of materials so that analytical characteristics are depicted. The phenomenon that native Chinese-speaking masters frequently repeat keywords of the thesis reflects the intuition-oriented mindset, highlighting the whole-to-part pattern and the inductive thinking model. The phenomenon that native English-speaking masters rarely repeat keywords of the thesis embodies the experience-oriented mindset, highlighting the part-to-whole pattern and the deductive thinking model.

With regard to distances between antecedents and anaphors set by native Chinese-speaking masters and native English-speaking masters, there are significant differences in the usage of distances among the four disciplines. No matter the Kurtosis or Skewness of distances, both values exceed the normal distribution value of 3 or 0. In statistics, if values of Kurtosis and Skewness are larger than normal distribution values, the histogram of distances definitely shows the features of the aiguille and fat tail branch.

According to Figure 1, there exist centered frequency distributions and large ranges of distance between antecedents and anaphors. Specifically, the number of words set between antecedents and anaphors by Chinese and foreign masters is controlled within a range of 0–50 words, but the average distance between antecedents and anaphors set by Chinese masters is 20.26 words, which is much longer than that set by foreign masters. The average distance set by foreign masters is merely 12.95 words. If the distance of 12.95 words is regarded as the distance threshold between antecedents and anaphors, the average distance set by Chinese masters exceeds this threshold.

## 5. Conclusion

The corpus is applied to compare and analyze the third personal pronoun endophora and its three elements in English abstracts of Chinese and foreign theses. Underlying reasons for similarities and differences are explored in order to help native Chinese-speaking masters have a better understanding of international writing conventions of English abstracts and to further improve the language quality of English abstracts in their theses.

In 480 English abstracts, there is no significant difference in the total frequency of third personal pronoun endophora used by native Chinese-speaking masters and native English-speaking masters. Driven by the economic principle of language, Chinese and foreign masters tend to avoid redundant words, reduce the memory burden of encoding and decoding, and finally improve the efficiency of language communication. Chinese masters pay attention to the cognitive schema from the whole to the part, and therefore the antecedents they use are usually consistent with keywords of the thesis. The direct repetition not only achieves the overall consistency of the thesis and the prominence of the theme, but also demonstrates the integrity and induction of the mindset. On the contrary, foreign masters show solicitude for the cognitive schema from the part to the whole, and hence the antecedents they apply are hardly consistent with the keywords of the thesis. The indirect description can not only lead readers to explore the whole topic when they experience different parts but also reflect the analytical and deductive mindset. Although the distance between antecedents and anaphors set by Chinese and foreign masters displays the same feature as the aiguille and fat tail branch, the distance set by Chinese masters far exceeds the threshold set by foreign masters. This finding has some implications for Chinese masters. When they use third personal pronoun endophora in English writing, they are suggested to shorten the distance between antecedents and anaphors in order to achieve discourse coherence.

It is concluded that native Chinese-speaking masters had better make efforts in terms of language representation and deep cognition in order to get closer to the international English abstract writing conventions. With regard to the language representation, Chinese masters are suggested to reduce the distance between antecedents and anaphors because the excessive distance will increase the memory burden of encoding and decoding for readers and have an influence on the readability and coherence of the discourse. In terms of deep cognition, 30 Chinese masters interviewed realize that they should pay attention to the cognitive schema of exploration and analysis and imitate the mindset of foreign masters. To be specific, the repetitiveness relationship between antecedents and keywords should be adjusted to the relevance relationship in order to comply with foreign masters' English abstract writing convention. Only the language representation and deep cognition are concerned, the language quality of English abstracts in their theses will be ultimately enhanced.

## Figures and Tables

**Figure 1:** Distances between antecedents and anaphors in CNKI and PQDT.

**Table 1:** Chi-square tests of third-personal pronoun endophora in CNKI and PQDT.

	Value	*df*	Asymp. Sig. (2-Sided)	Exact sig. (2-sided)	Exact sig. (1-sided)
Pearson Chi-square	0.055a	1	0.815		
Continuity correction^b^	0.020	1	0.889		
Likelihood ratio	0.054	1	0.816		
Fisher's exact test				0.852	.443
Linear-by-linear association	0.055	1	0.815		
*N* of valid cases	2281				

a. 0 cells (0.0%) have an expected count of less than 5. The minimum expected count is 51.75. b. Computed only for a 2 × 2 table.

**Table 2:** Multivariate tests^b^ of three elements of third personal pronoun endophora in CNKI and PQDT.

Effect		Value	*F*	Hypothesis *df*	Error *df*	Sig.
Intercept	Pillai's trace	0.962	13684.131^a^	3.000	2152.000	0.000
	Wilks' lambda	0.038	13684.131^a^	3.000	2152.000	0.000
	Hotelling's trace	25.435	13684.131^a^	3.000	2152.000	0.000
	Roy's largest root	25.435	13684.131^a^	3.000	2152.000	0.000

Source	Pillai's trace	0.066	38.061^a^	3.000	2152.000	0.000
	Wilks' lambda	0.934	38.061^a^	3.000	2152.000	0.000
	Hotelling's trace	0.071	38.061^a^	3.000	2152.000	0.000
	Roy's largest root	0.071	38.061^a^	3.000	2152.000	0.000

a. exact statistic and b. design: intercept + source.

## Data Availability

No data were used to support this study.
